This article has been retracted.

# The Akt inhibitor KP372-1 suppresses Akt activity and cell proliferation and induces apoptosis in thyroid cancer cells

**DOI:** 10.1038/sj.bjc.6602595

**Published:** 2005-05-03

**Authors:** M Mandal, S Kim, M N Younes, S A Jasser, A K El-Naggar, G B Mills, J N Myers

**Affiliations:** 1 Department of Head and Neck Surgery, The University of Texas MD Anderson Cancer Center, Houston, TX, USA; 2 Department of Pathology, The University of Texas MD Anderson Cancer Center, Houston, TX, USA; 3 Department of Molecular Therapeutics, The University of Texas MD Anderson Cancer Center, Houston, TX, USA

**Keywords:** molecular therapy, growth factors, anaplastic thyroid cancer, KP372-1

## Abstract

The phosphatidylinositol 3′ kinase (PI3K)/phosphatase and tensin homologue deleted on chromosome ten/Akt pathway, which is a critical regulator of cell proliferation and survival, is mutated or activated in a wide variety of cancers. Akt appears to be a key central node in this pathway and thus is an attractive target for targeted molecular therapy. We demonstrated that Akt is highly phosphorylated in thyroid cancer cell lines and human thyroid cancer specimens, and hypothesised that KP372-1, an Akt inhibitor, would block signalling through the PI3K pathway and inhibit cell proliferation while inducing apoptosis of thyroid cancer cells. KP372-1 blocked signalling downstream of Akt in thyroid tumour cells, leading to inhibition of cell proliferation and increased apoptosis. As thyroid cancer consistently expresses phosphorylated Akt and KP372-1 effectively blocks Akt signalling, further preclinical evaluation of this compound for treatment of thyroid cancer is warranted.

The incidence of thyroid cancer in the United States is expected to be approximately 23 600 in 2004 (Jemal *et al*, 2004). Thyroid carcinomas can be classified into papillary thyroid carcinoma, follicular thyroid carcinoma, and anaplastic thyroid carcinoma (Jemal *et al*, 2004). The papillary and follicular thyroid carcinomas constitute the majority of thyroid carcinomas and are grouped together as well-differentiated thyroid carcinomas. This group of thyroid carcinomas can often be cured with surgical resection and with radioactive iodide therapy. However, there are no effective alternative therapies for patients with metastatic well-differentiated thyroid cancer who do not respond to radioactive iodine therapy, suggesting an urgent need for development of novel therapies.

The pathogenesis of thyroid cancer is characterised by the alterations of multiple signalling pathways and by abnormalities in a variety of tumour-suppressor genes and cell-cycle proteins (Fagin, 2002). The activation of the Akt protein kinase B (Akt/PKB) signalling pathway appears to play an important role in the development and progression of thyroid tumours. Interestingly, Akt has been found to be activated by a genetic loss of expression of phosphatase and tensin homologue deleted on chromosome ten (PTEN), a tumour-suppressor gene, in Cowden's syndrome, an autosomal dominant multi-organ hamartoma syndrome characterised by benign and malignant thyroid tumours and breast and colon cancers (Dahia *et al*, 1997; Liaw *et al*, 1997). Akt activation, probably through a variety of mechanisms including aberrant stimulation of upstream cancers, occurs in most sporadic thyroid cancers (Ringel *et al*, 2001). In benign thyroid cell models, Akt signalling is important for cell growth in response to insulin, insulin-like growth factor-1, and serum (Kimura *et al*, 1999, 2001; Coulonval *et al*, 2000; Saito *et al*, 2001) and is activated by several oncogenes involved in thyroid cancer, including activated *p21*^*ras*^ and chimeric rearrangements involving the *ret* gene (*RET/PTC* oncogenes) (Borrello *et al*, 1994; Rodriguez-Viciana *et al*, 1994). Despite the central role for Akt activation in thyroid tumorigenesis, little is known about the biological effect of inhibition of the Akt kinase in the progression of thyroid carcinoma.

Based on the putative central role of the Akt kinase in thyroid oncogenesis, we hypothesised that KP372-1, a specific Akt kinase inhibitor (molecular weight, 224.20; QLT Inc., Vancouver, BC, Canada), would inhibit the proliferation and induce apoptosis of thyroid cancer cells *in vitro*. KP372-1 was identified in a screen of kinase-inhibiting compounds tested on more than 100 different cellular kinases, and was selected for its high specificity for the Akt kinase (unpublished data from QLT). In this study, we demonstrated the key role of the phosphatidylinositol-3 kinase (PI3K)/Akt pathway in thyroid cancer and explored the effect of KP372-1 using thyroid cancer cells as model systems. We assessed the effects of KP372-1 on the inhibition of the PI3K/Akt pathway biochemically and on cell proliferation and apoptosis.

## MATERIALS AND METHODS

### Cell lines

A papillary thyroid carcinoma cell line, NPA187, a follicular thyroid cancer cell line, WRO, and anaplastic thyroid cancer cell lines KAT4, C643, K18, HTH74, ARO, and DRO were used. NPA187 and WRO were obtained from Dr Yan Oh, The University of Texas MD Anderson Cancer Center, Houston, TX, USA, and KAT4, C643, K18, HTH74, and DRO were obtained from Dr Sai-Ching Jim Yeung, Department of Endocrine Neoplasia and Hormonal Disorders, MD Anderson Cancer Center, Houston, TX, USA. All the cell lines were grown in RPMI medium supplemented with 10% foetal bovine serum, L-glutamine, penicillin, sodium pyruvate, nonessential amino acids, and vitamin solution (Life Technologies, Inc., Grand Island, NY, USA). Adherent monolayer cultures were maintained on plastic and incubated at 37°C in 5% carbon dioxide and 95% air. The cultures were free of *Mycoplasma* species. The cultures were maintained no longer than 12 weeks after recovery from frozen stocks.

### Compounds

KP372-1 (Figure 1) was synthesised by QLT Inc., Vancouver, BC, Canada. KP372-1 is a mixture of two isomers present in approximately equal amounts. A stock solution of KP372-1 for enzyme or cellular assays was prepared in dimethyl sulphoxide (DMSO) and then diluted in the medium. The final concentration of DMSO in the incubation mixture did not exceed 0.1% v v^−1^.

### Tissue samples and Western blotting

Fresh frozen human thyroid tissue specimens were obtained from the thyroid tissue bank (The University of Texas MD Anderson Cancer Center) with the approval of the Institutional Review Board at the MD Anderson Cancer Center. Thyroid specimens from patients who had undergone surgery were carefully harvested by an experienced pathologist (AKE) and were snap frozen in liquid nitrogen and stored at −80°C. Thawed tissue samples were homogenised in Triton X-100 lysis buffer (20 mM HEPES, 50 mM NaCl, 1% Triton X-100, 0.1% deoxycholate, 2 mM EDTA, 2 mM sodium vanadate, and protease inhibitor cocktail), and equal amounts of protein were analysed by Western blotting. The following antibodies were used for Western blotting: rabbit anti-pAkt (S473), rabbit anti-pAkt (T308), and rabbit anti-Akt (Cell Signaling, Beverly, MA, USA), rabbit anti-p85 and rabbit anti-PTEN (Santa Cruz, Santa Cruz, CA, USA), and rabbit anti-*β*-actin (Sigma, St Louis, MO, USA). *β*-Actin was used as a loading control.

### Cell proliferation

For MTT assays involving treatment with KP372-1, the cells were diluted to 1000 cells per 100 *μ*l of complete medium, from which 100 *μ*l was added to each well of a 96-well plate (Falcon; Becton-Dickinson, Franklin Lakes, NJ, USA). On the following day, 100 *μ*l of medium supplemented with two times the desired concentration of KP372-1 was added to the appropriate wells. The cells were then kept at 37°C in 5% CO_2_ for 72 h. At this point, 10 *μ*l of a 5 mg ml^−1^ stock solution of MTT (Sigma) dissolved in water was added to each well, and the plates were returned to the 37°C incubator for 2 h. The supernatant was aspirated out of each well, and 200 *μ*l of DMSO was added to each well. The plates were then shaken for 5 min and the optical density measured at 570 nm using a spectrophotometer.

To measure the cell proliferation, we plated the NPA187 and WRO cells at a concentration of 1 × 10^4^ cells well^−1^ in six-well plates. The cells were then treated with KP372-1 at a concentration of 30 and 60 nM for NPA187 and WRO cell lines, respectively, and were counted using a haemocytometer on days 1, 2, and 3.

### ^3^H-thymidine incorporation

DNA synthesis in the control and KP372-1-treated cells was assessed by the incorporation of ^3^H-thymidine into newly replicated DNA. NPA187 and WRO cells were plated at a concentration of 5000 cells well^−1^ in 96-well plates. After 24 h, the cells were treated with different concentrations of KP372-1 for 48 h and treated with 5-*μ*Ci ml^−1^ ^3^H-thymidine during the last 2 h (NEN Life Science Products, Inc., Boston, MA). Cells were washed with PBS and then extracted with 0.1 N KOH and counted by liquid scintillation.

### DNA fragmentation assay

For the DNA fragmentation assay, low-molecular-weight DNA was prepared (Mandal *et al*, 1996). Briefly, NPA187 and WRO cells (3 × 10^6^ per plate) were seeded in 100 mm plates and treated with KP372-1 (30 nM for NPA187 and 60 nM for WRO) for 1, 2, or 3 days. Both floating and attached cells were scraped and collected in medium, washed three times with PBS, and resuspended in 1 ml of lysis buffer (20 mM Tris-HCl (pH 8), 10 mM EDTA (pH 8), and 0.5% Triton X-100). After incubation on ice for 30 min, the lysates were spun at 12 000 rpm in a microcentrifuge for 10 min. Low-molecular-weight DNA in the supernatant was extracted with equal volumes of phenol and chloroform for 1 h at 4°C. Ammonium acetate (2 M) was added to the aqueous phase, and the DNA was precipitated with two volumes of ethanol at −20°C overnight. The DNA was treated with RNAse A (1 mg ml^−1^) at 37°C for 1 h, and total DNA was analysed using 1.5% agarose gel and visualised with ethidium bromide staining.

### Western blot analysis of thyroid carcinoma cell lines after treatment with KP372-1

In order to show the induction of apoptosis-related proteins by KP372-1, NPA187 and WRO cells (3 × 10^6^ per plate) were seeded in 100 mm plates and treated with KP372-1 (30 nM for NPA and 60 nM for WRO) for 1, 2, or 3 days. Both floating and attached cells were scraped and collected in medium, washed three times with PBS, and the cells were lysed in Nonidet P-40 lysis buffer (50 mM Tris-HCl (pH 8.0), 137 mM NaCl, 10% glycerol, 1% Nonidet P-40, 50 mM NaF, 10 mM *β*-glycerol phosphate) containing 1 mM sodium vanadate, 1 mM phenylmethylsulphonyl fluoride, 10 *μ*g ml^−1^ apoptinin, and lysis buffer (20 mM Tris-HCl (pH 8), 10 mM EDTA (pH 8), and 0.5% Triton X-100). After incubation on ice for 30 min, the lysates were spun at 12 000 rpm in a microcentrifuge for 10 min. Equal amounts of protein were then analysed by Western blotting using the following antibodies: mouse anti-poly(ADP-ribose)polymerase (PARP) antibody (Trevigen, Gaithersburg, MD, USA), rabbit anti-caspase-3 antibody (Cell Signaling), and rabbit anti-*β* actin antibody (Sigma). *β*-Actin was used as a loading control.

In order to show the effect of KP372-1 on various signal transduction pathways in thyroid carcinoma cell lines, we performed Western blot analysis on NPA187 and WRO cells after treating the cells with KP372-1. The cells were plated as described above. After treating the cells with KP372-1 (30 nM for NPA187 and 60 nM for WRO) for 4 h, both floating and attached cells were scraped and collected in medium, washed three times with PBS, and lysed with a lysis buffer as described above. After incubation on ice for 30 min, the lysates were spun at 12 000 rpm in a microcentrifuge for 10 min. Equal amounts of protein were then analysed by Western blotting using the following antibodies: rabbit anti-pAkt (S473), rabbit anti-Akt, rabbit anti-p-mitogen-activated protein kinase (MAPK), rabbit anti-pmTOR, rabbit anti-pS6R, and rabbit anti-S6R (Cell Signaling).

### Akt enzyme assay to detect *in vitro* kinase activity

Cells were lysed using the lysis buffer provided in the Akt enzyme assay kit (Cell Signaling). The cells were scraped and placed in an Eppendorf centrifuge tube incubated on ice for 15 min and spun in a centrifuge at 4°C for 15 min at full speed. The lysates were then transferred to a new tube and stored at −80°C until assayed.

Immunoprecipitation was carried out as follows: 500 *μ*g of protein was added to 5 *μ*l of anti-Akt antibody (Cell Signaling) and rotated at 4°C overnight. Protein A sepharose beads (50 *μ*l) were then added and rotated for 3 h at 4°C. The protein A sepharose beads were then washed three times with lysis buffer and three times with the 1 × kinase buffer provided in the kit. Then the beads were aspirated, and 40 *μ*l of kinase buffer was supplemented with 200 *μ*M ATP and a mixture (1 *μ*g per 40 *μ*l) of fusion protein (provided in the kit). The tubes were then incubated at 30°C for 30 min, after which 20 *μ*l of 3 × sample buffer consisting of 187.5 mM Tris-HCl (pH 6.8), 6% (w v^−1^) sodium dodecyl sulphate (SDS), 30% glycerol, 150 mM DTT, and 0.03% (w v^−1^) bromophenol blue was added to each tube. The tubes were then boiled for 5 min at 95°C, and glycogen synthetase kinase-3 (GSK-3) phophorylation was measured using phospho antibodies (Cell Signaling).

## RESULTS

### Akt is phosphorylated in many thyroid cancer cell lines

In an attempt to delineate the role of Akt signalling in thyroid cancer cells, we first profiled the expression of pAkt, total Akt, and the p85 subunit of PI3K in a panel of thyroid cancer cell lines. As seen in Figure 2, most thyroid cancer cell lines expressed readily detectable levels of pAkt-Ser473, pAkt-Thr308, total Akt, and subunits of the PI3K p85. PTEN was present in all the cell lines. The low levels of pAkt in some cell lines was likely due to the relative levels of pAkt rather than complete absence of this molecule. Three cell lines were selected for further characterisation: NPA187, which expressed relatively high levels of pAkt, and total Akt, K18, which expressed high levels of pAkt and low levels of total Akt, and WRO, which expressed lower levels of pAkt with high levels of total Akt. The presence of similar amounts of PTEN (most mutant PTEN molecules are unstable) in these cell lines suggests that the difference in pAKT levels was likely not due to defective PTEN function.

### Akt expression in human thyroid cancer tissues

After profiling the expression of Akt and pAkt in thyroid cancer cell lines, we focused our attention on the role of Akt in well-differentiated thyroid carcinoma in subsequent experiments. To determine whether our *in vitro* findings with cell lines reflected the biology of human thyroid cancer *in vivo*, we evaluated the expression of Akt and pAkt in fresh papillary thyroid tumour specimens using Western blotting. The status of Akt activation was examined using a phosphorylation-specific antibody against pAkt-Ser473 and antibody against total Akt in thyroid tumours and adjacent normal-appearing tissues. As shown in Figure 3, six of eight tumours had higher levels of phosphorylated Akt-Ser473 than did normal tissues despite similar levels of total Akt. Akt phosphorylation was higher in the thyroid tumours than in the neighbouring normal tissues, suggesting a potential role for Akt phosphorylation in the carcinogenesis of thyroid cancer. The high levels of Akt phosphorylation in neighbouring tissue samples from some patients may reflect a ‘field effect’ due to genetic aberrations or, alternatively, the production and action of paracrine growth factors by the tumours.

### KP372-1 inhibits proliferation and induces the apoptosis of thyroid cancer cells *in vitro*

The effect of KP372-1 on the growth of NPA187 and WRO cells was evaluated using an MTT assay, cell counting, and ^3^H-thymidine incorporation. The proliferation of these cell lines was inhibited by KP372-1 with an IC_50_ (concentration at which 50% inhibition occurs) of 30 and 60 nM for NPA187 and WRO, respectively (Figure 4). The proliferation of the cell lines was also inhibited by KP372-1, as evidenced by cell counting (Figure 5A and B) and the ^3^H-thymidine incorporation assay (Figure 5C and D). As shown in Figure 2, different levels of pAkt and total Akt were seen in the three cell lines. As shown in Figure 4, the NPA187 cell line, which had high basal pAkt levels, was more sensitive to KP372-1 than was WRO, which had low pAkt levels, suggesting that high pAkt could indicate cell dependence on this pathway and thus higher sensitivity to the inhibition of Akt.

This decreased MTT incorporation can be due to a decreased rate of cell cycle transit or increased cell death. To assess the latter possibility, we treated the NPA187 and WRO cells with KP372-1 for different lengths of time and determined the extent of apoptosis by DNA fragmentation (Figure 6A) and the accumulation of a sub-G_0_/G_1_ cell population by flow cytometry (data not shown). The effect of KP372-1 on the status of PARP and caspase-3 was also examined (Figure 6B). The induction of activated caspase-3 and cleavage of PARP by KP372-1 treatment were observed in both cell lines, although with different kinetics and different magnitudes. Consistent with the MTT data, NPA187 demonstrated greater degrees of PARP cleavage and DNA degradation at 72 hours than WRO.

To determine the duration of exposure to KP372-1 required to commit cells to apoptosis, NPA187 and WRO cells were incubated with 30 and 60 nM of KP372-1, respectively, for 6 h in serum-free medium. The cells were then washed with PBS and grown in medium containing 10% FBS without the inhibitor for another 24 or 48 h. The cells were then assayed for the percentage of apoptotic cell death. Apoptosis was not induced under these conditions (data not shown). Thus, we concluded that KP372-1 must be present continuously in order to induce apoptosis at least at these doses and for these cell lines.

### KP372-1 inhibits Akt kinase activity, phosphorylation of Akt, and downstream targets of Akt in thyroid cancer cells

We next determined the effect of KP372-1 on the phosphorylation of AKT (Ser473) and on downstream targets of Akt, including p-mTOR and p-S6 ribosomal protein (Ser240/244), and MAPK. We treated NPA187 and WRO cells with KP372-1 at their respective IC_50_ for 4 h and analysed the cell lysates with the specific antibodies indicated in Figure 7A. In the case of NPA187 and WRO, phosphorylation of Akt and S6 ribosomal protein was downregulated by treatment with KP372-1. However, the phosphorylation of mTOR and MAPK was not changed by treatment with KP372-1. Akt kinase activity was also downregulated by KP372-1 in multiple thyroid cancer cell lines, as tested by an *in vitro* kinase assay using GSK-*β* as substrate (Figure 7B).

Our results indicate that KP372-1 blocks Akt kinase activity, thereby decreasing phosphorylation of the S6 ribosomal protein. The mechanism resulting in the decrease in Akt phosphorylation is under exploration, but may represent an allosteric change in the molecule, decreasing access to upstream kinases or increasing access to downstream phosphatases.

## DISCUSSION

Our study shows that thyroid cancer cells expressed detectable levels of Akt Ser473, Akt-Thr308, total Akt, PTEN, and the p85 subunits of the PI3K and Akt kinase activity. Most of the tumours showed a higher level of Akt-Ser473 phosphorylation than matching normal tissues, suggesting an association between a high level of Akt phosphorylation and thyroid carcinogenesis. This association was further supported by evidence that blockade of Akt signalling with the selective inhibitor KP372-1 induced apoptosis and inhibited cell proliferation in human thyroid cancer cell lines in culture. Furthermore, KP372-1 was found to inhibit the phosphorylation and kinase activities of Akt in addition to the phosphorylation of downstream substrates. However, the mechanism responsible for decreased Akt phosphorylation is not clear. It is possible that the binding of KP372-1 to Akt may alter its conformation so that the relevant amino-acid residues are not available for phosphorylation. A similar effect has been seen with other inhibitors such as those for MEK1 and JNK where they decrease phosphorylation of their target in cells with an activated pathway.

In our study, we found that the papillary thyroid cancer cell line NPA187 was more sensitive to the effects of KP372-1 compared with the follicular cell line WRO. However, Ringel *et al* (2001) found that the cell line NPA187 was more sensitive than WRO to the effects of LY294002, a phosphatidylinositol 3′ kinase (PI3K) inhibitor. This difference in sensitivities to two different agents that target the same pathway may be due to the fact that these agents show affinity for kinases other than the intended primary target kinase. It is also known that KP372-1 inhibits kinases other than Akt, such as CDK1, CK2, CSK, DNAPK, ERK1, GSK3b, LCK, MEK1, PIM, PKA, PKC, and S6K, albeit at relatively high concentrations (unpublished work from QLT). We have also found that the NPA187 cell line showed higher levels of Akt phosphorylation than WRO. This observation suggests that NPA187 may be more dependent than WRO on the activation of Akt for survival and proliferation.

Inhibition of Akt might be of great benefit to patients with aggressive thyroid cancers, and support for the concept of targeting Akt comes from many observations. First, more than 54% of human cancers have active Akt that is detectable *in situ* (Bellacosa *et al*, 1991). Akt activation was identified in 10 of 10 follicular cancers, 26 of 26 papillary cancers, and two of 10 follicular variants of papillary cancers, but in only four of 66 normal tissue samples and two of 10 typical benign follicular adenomas (Vasko *et al*, 2004). Second, pAkt expression was found to be greatest in regions of capsular invasion and was localised to the nucleus in follicular cancers and to the cytoplasm in papillary cancers, except for invasive regions of papillary cancers, where it localised to both compartments (Vasko *et al*, 2004). Thus, small-molecule Akt inhibitors could have wide applicability as anticancer drugs. Third, inhibition of the PI3K/Akt pathway by biochemical or genetic means increases the efficacy of chemotherapy, radiotherapy, or both, *in vitro* and *in vivo* (Hu *et al*, 2000; Brognard *et al*, 2001; Bondar *et al*, 2002). Finally, several standard chemotherapeutic and chemopreventive agents inhibit the PI3K/Akt pathway when administered *in vitro*, and, in some cases, inhibition of Akt is directly responsible for these agents' cytotoxicity (West *et al*, 2002).

Despite the acknowledged need for Akt inhibitors, none is widely available and none that inhibits the kinase activity of Akt is in clinical evaluation. The current studies indicate that KP372-1 acts to inhibit Akt and has activity in cells with high levels of pAkt. This is similar to other inhibitors of the PI3K/Akt pathway, such as Wortmannin and LY294002. Wortmannin and LY294002 may have limited clinical utility because they lack specificity and have potential adverse side effects, poor pharmacological properties, low stability, and poor solubility (West *et al*, 2002). Wortmannin inhibits myosin light-chain kinase; phospholipases C, D, and A_2_; and DNA-dependent protein kinase (West *et al*, 2002). LY294002 also inhibits the aryl hydrocarbon receptor, a ligand-activated transcription factor (Guo *et al*, 2000). *In vivo* use of LY294002 in mice has been associated with many adverse effects, including death (Hu *et al*, 2002). Similarly, Wortmannin has demonstrated hepatic and haematopoietic toxicity. Therefore, although Wortmannin and LY294002 inhibit the PI3K/Akt pathway, their drawbacks raise doubts about their suitability as leading candidates for additional development.

The major advantage of KP372-1 over Wortmannin and LY294002 as PI3K inhibitors is its greater efficacy and the marked induction of apoptosis in cancer cell lines. This may be due to its targeting a central downstream molecule and also due to the potential for a number of processes to bypass effects at the level of PI3K. However, the final determination will be in terms of therapeutic index, which will need to be evaluated in mice and eventually humans. Indeed, a potential downside of Akt inhibitors is toxicity because of the importance of Akt signalling in many normal cellular processes such as insulin signalling, and the lack of selectivity of the current Akt inhibitors including KP372-1 to different Akt isoforms. Identifying kinase inhibitors that target the ATP-binding site of a kinase can be fraught with specificity problems because all kinases and many other molecules possess ATP-binding sites. This was perhaps best observed with STI-571 (Gleevec, imatinib mesylate, Novartis Pharma, Basel, Switzerland), a competitive inhibitor of the ATP-binding site of many kinases (Klejman *et al*, 2002). The wide clinical application of STI-571 is partially due to its ability to inhibit many kinases, including bcr–abl, platelet-derived growth factor receptors, and c-Kit (Heinrich *et al*, 2000; McGary *et al*, 2002; von Bubnoff *et al*, 2002). The relatively nonspecific activity of STI-571 results in activity against Kit and the PDGFR in gastrointestinal stromal tumours (GIST) and against the PDGFR in hypereosinophilic syndrome. It is somewhat surprising and fortuitous that the relative broad activity of STI-571 was not associated with toxicity.

In conclusion, thyroid cancer cell lines and well-differentiated human tumour specimens showed high levels of Akt phosphorylation on Ser473 and high Akt activity levels, which supported the findings of several other studies (Dahia *et al*, 1997; Liaw *et al*, 1997; Ringel *et al*, 2001), indicating that the Akt signalling pathway plays a role in thyroid cancer progression. In addition, specific inhibition of Akt kinase activity by KP372-1 resulted in decreased cell proliferation and induction of apoptosis of thyroid cancer cells *in vitro*. Although anaplastic thyroid cell lines were included in some of our experiments, our data lend support to the use of Akt kinase inhibitor in well-differentiated thyroid carcinoma rather than in anaplastic or poorly differentiated thyroid carcinomas. These findings indicate that further preclinical evaluation of this and other compounds targeting the PI3K/Akt pathway in well-differentiated thyroid cancer is warranted.

## Figures and Tables

**Figure 1:** Molecular structure of KP372-1.

**Figure 2:** Expression of phosphorylated (p) Akt-Ser473, pAkt-Thr308, p85, subunits of PI3K, and PTEN in thyroid cancer cell lines. Cell lysates from exponentially growing cells were analysed by immunoblotting with antibodies against the indicated proteins. Results shown are representative of three independent experiments.

**Figure 3:** Akt expressions in human thyroid cancer. Expression of pAkt (Ser473) and total Akt in thyroid tumours (T) and adjacent normal tissues (N) were detected with immunoblotting.

**Figure 4:** Effects of KP372-1 on the proliferation of thyroid carcinoma cell lines *in vitro*. Thyroid carcinoma cell lines NPA187 and WRO were plated in a 96-well plate and treated with different concentrations of KP372-1 for 48 h. Cell growth was measured by MTT assay. Results shown are representative of three experiments.

**Figure 5:** Effects of KP372-1 on the proliferation of thyroid carcinoma cell lines *in vitro*. (**A**, **B**) Thyroid carcinoma cell lines NPA187 and WRO were plated in six-well plates and treated with 30 and 60 nM KP372-1 for NPA187 and WRO cell lines, respectively, for 1, 2, or 3 days. Cell proliferation was then measured by cell counting using a haemacytometer. (**C**, **D**) Thyroid carcinoma cell lines NPA187 and WRO were plated in a 96-well plate and treated with various concentrations (0–120 nM) of KP372-1 for 48 h. Cell proliferation was then measured by ^3^H-thymidine incorporation. Results shown are representative of three experiments.

**Figure 6:** KP372-1 induces apoptosis in thyroid cancer cells *in vitro*. (**A**) Cells were treated with KP372-1 as indicated for various periods. DNA fragmentation was measured by ethidium bromide staining after the DNA was resolved on an agarose gel. (**B**) Cells were treated with KP372-1 for different time periods, and cell extracts were immunoblotted with the indicated antibodies. Results shown are representative of three experiments with similar results.

**Figure 7:** KP372-1 inhibits Akt phosphorylation and some of the downstream signalling molecules as well as Akt kinase activity. (**A**) NPA187 and WRO cells were treated with the IC_50_ concentrations of KP372-1 (30–60 nM, respectively) for 4 h in RPMI medium without serum. Equal amounts of protein were resolved by SDS–polyacrylamide gel electrophoresis and immunoblotted with different antibodies as indicated. (**B**) KP372-1 inhibits Akt kinase activity. Different thyroid cancer cells were treated with KP372-1 for 2 h, cell lysates were prepared, and Akt was immunoprecipitated and analysed for Akt-Ser473 and Akt kinase activity using an *in vitro* kinase assay with GSK-*β* as a substrate. Results shown are representative of three experiments.
